The article "Peroneal Electric Transcutaneous NeuroModulation (eTNM®): A Novel Method for the Treatment of the Overactive Bladder" was published in 2021. Journal: J Healthc Eng.

# Peroneal Electric Transcutaneous NeuroModulation (eTNM^®^): A Novel Method for the Treatment of the Overactive Bladder

**DOI:** 10.1155/2021/4016346

**Published:** 2021-10-06

**Authors:** Jan Krhut, Lukas Peter, Michal Rejchrt, Martin Slovak, Barbora Skugarevska, Peter Zvara

**Affiliations:** ^1^Department of Urology, University Hospital, Ostrava, Czech Republic; ^2^Department of Surgical Studies Medical Faculty, Ostrava University, Ostrava, Czech Republic; ^3^STIMVIA™, Ostrava, Czech Republic; ^4^Department of Chemistry Faculty of Science, University of Hradec Králové, Hradec Králové, Czech Republic; ^5^Department of Urology, 2nd Faculty of Medicine of Charles University and Motol University Hospital, Prague, Czech Republic; ^6^Biomedical Laboratory and Research Unit of Urology Department of Clinical Research, University of Southern Denmark, Odense, Denmark; ^7^Department of Urology, Odense University Hospital, Odense, Denmark

## Abstract

Overactive bladder syndrome (OAB) is a prevalent medical problem with a significant impact on the quality of life of the affected individuals. Pharmacotherapy is considered the main treatment method, although it is discontinued in a significant proportion of patients due to inefficacy or associated side effects. If pharmacotherapy fails, patients can undergo peripheral neuromodulation of the somatic nerves of the lower limb or sacral neuromodulation; however, neither of these represents an ideal therapeutic tool. The Peroneal electric Transcutaneous NeuroModulation (Peroneal eTNM^®^), based on the selective stimulation of the peroneal nerve, is the new fully noninvasive neuromodulation method intended to treat OAB. The URIS^®^ neuromodulation system, engineered to provide Peroneal eTNM^®^, consists of the URIS^®^ device, URIS^®^ active electrodes, and the biofeedback foot sensor (BFS). The unique design of the URIS^®^ device and URIS^®^ active electrodes allows for the use of a low voltage and current during neuromodulation, which significantly reduces the unpleasant sensations. The BFS allows for precise localization of the active electrodes and for continuous adjustment of the voltage and frequency to achieve the optimal therapeutic effect. The URIS^®^ system adopts several principles of telemedicine, which makes it compatible with the US Food and Drug Administration (FDA) and European Union (EU) regulations for home-based use. This article describes both the Peroneal eTNM^®^ method and the URIS^®^ neuromodulation system, including its technical specifications and data from laboratory testing. Preclinical and early clinical data demonstrate the feasibility of this new method for noninvasive OAB treatment and possible implications for clinical practice.

The article "Peroneal Electric Transcutaneous NeuroModulation (eTNM®): A Novel Method for the Treatment of the Overactive Bladder" was published in 2021. Journal: J Healthc Eng.

## 1. Introduction

Overactive bladder syndrome (OAB) represents lower urinary tract dysfunction; it is a sudden, compelling desire to pass urine that is difficult to defer (urgency), with or without involuntary loss of urine associated with the urgency (urgency urinary incontinence) [1]. A significant proportion of patients with OAB also suffer from frequent voiding (frequency) and getting up at night to pass urine (nocturia) [2]. OAB represents one of the most common urological problems, affecting 10.8–16.9% of the adult population worldwide [3]. OAB has a significant impact on quality of life (QoL), employment, social status, and relationships [4].

Initial conservative treatment includes lifestyle interventions, behavioral techniques, and pelvic floor muscle exercises. Pharmacotherapy is the most widely used treatment method. However, its efficacy is insufficient in at least 30% of patients [5]. In addition, its use is often associated with unacceptable systemic side effects that often lead to the discontinuation of treatment. Although the persistence rates for OAB medication improved with the introduction of mirabegron, recent studies showed that the 12-month persistence is 24–41% [6]. According to the current clinical guidelines, peripheral neuromodulation of the somatic nerves of the lower limb or sacral neuromodulation can be offered to the patients who failed previous first-line therapy [7]. Percutaneous tibial nerve stimulation (PTNS) is the most widely used peripheral neuromodulation method for the treatment of OAB in clinical practice [8]. The main disadvantage of PTNS is the need to insert a 34-gauge needle electrode close to the tibial nerve, which is usually uncomfortable or painful to patients and requires some skills. This is why PTNS is mostly performed in outpatient settings by trained medical staff, thus increasing the costs and limiting availability [9].

Given these limitations, surface electrodes were introduced to deliver impulses to the tibial nerve in transcutaneous tibial nerve stimulation (TTNS) [10]. TTNS showed some benefits in terms of alleviating OAB symptoms [11]. However, there are several limitations of TTNS, including an absence of standardization of the position of the electrodes, leading to inconsistent nerve activation, and the use of large surface electrodes, causing significant spread of electrical field in the tissue that results in poor electrical recruitment of deep nerves. All these factors may deteriorate the clinical effect [12].

Given that neuromodulation may represent a causal treatment for at least a certain proportion of OAB patients, the development of a new method that would address the limitations of both PTNS and TTNS is highly desirable.

The article "Peroneal Electric Transcutaneous NeuroModulation (eTNM®): A Novel Method for the Treatment of the Overactive Bladder" was published in 2021. Journal: J Healthc Eng.

This paper includes a description and critical evaluation of a new fully noninvasive neuromodulation method called Peroneal electric Transcutaneous NeuroModulation (Peroneal eTNM^®^) that is intended to treat the OAB syndrome.

## 2. Method Description

The basic principle of the Peroneal eTNM^®^ is based on the use of electrical impulses to activate the afferent fibers of the peroneal nerve, which affects the neural structures involved in the control of the urinary bladder. The peroneal nerve represents one of the two main branches of the sciatic nerve and contains nerve fibers originating from the lumbar spinal segments L4-L5 and the sacral spinal segments S1–S2. Motor fibers of the peroneal nerve innervate the skeletal muscles at anterior and lateral aspects of the leg, while sensory fibers supply the dermatomes at the lateral aspect of the leg and the dorsal aspect of the foot [13]. After separation from the sciatic nerve, the peroneal nerve runs laterocaudally along the inner edge of the biceps femoris muscle. At the level of the popliteal fossa, the nerve is covered by the skin, fascia, and adipose tissue, but not by the muscle as shown in Figure 1.

The Peroneal eTNM^®^ using the URIS^®^ neuromodulation system could be delivered in a supine or sitting position. The URIS^®^ active electrodes are placed bilaterally directly on the skin over the lateral part of the popliteal fossa in the proximity of the medial aspect of the biceps femoris muscle. A self-adhesive neutral electrode is placed on the lower abdomen, closing the stimulation circuit for both active electrodes. After setting the initial frequency to 4 Hz and voltage to 20 V, the optimal stimulation point (OSP) is detected using the discrete corrections of the electrode position. The OSP is an area of about 0.8 cm^2^ and can be localized based on eliciting both sensation and visible motor response characterized by rhythmic lateromedial foot movement (Figure 2). Once the OSP is set, the voltage is adjusted to the lowest value eliciting a motor response, and the neuromodulation session is initiated. The treatment strategy includes a 30-minute session once a week for 12 weeks.

Our understanding of the mechanism of action of Peroneal eTNM^®^ is based mostly on evidence of a connection between somatic innervation of the lower limbs and autonomic innervation of the pelvic organs. These connections affect autonomic bladder innervation by selective neuromodulation of the afferent somatic nerve fibers originating from the same spinal cord segments [14]. Some animal studies indicate that neuromodulation of the nerves originating from the sacral spinal cord affects the supraspinal centers and regulatory circuits involved in the control of the lower urinary tract [15]. These data suggest that the effect of Peroneal eTNM^®^ on bladder function might involve various mechanisms at several levels of the neural control.

The article "Peroneal Electric Transcutaneous NeuroModulation (eTNM®): A Novel Method for the Treatment of the Overactive Bladder" was published in 2021. Journal: J Healthc Eng.

## 3. Neuromodulation System Description

The novel URIS^®^ neuromodulation system (STIMVIA™, Ostrava, Czech Republic, EU) designed to provide Peroneal eTNM^®^ consists of the URIS^®^ device, specially engineered URIS^®^ active electrodes, and the biofeedback foot sensor (BFS).

### 3.1. URIS^®^ Device

This device consists of the impulse generator, which is controlled by the microcontroller unit (MCU). The MCU has its own hardware (HW) periphery and firmware. Unlike the other generators currently used for PTNS and TTNS, the URIS^®^ generator is designed as a voltage source. The generator provides impulses with a primarily monophasic rectangular waveform; the voltage amplitude is adjustable, in the range of 0–90 V, the frequency range is 0–10 Hz, and the impulse width is 2 ms. After the impulse time has elapsed, the patient is electronically disconnected from the electric circuit completely. The electrical safety of the URIS^®^ device was tested under the IEC 60601-1 and IEC 60601-2-10 requirements.

### 3.2. URIS^®^ Active Electrodes

Electrical impulses are delivered to the patient's body through the active electrodes connected to the device. The electrode was designed to allow for selective stimulation of the individual nerve (similar to the needle electrode) while maintaining simple and noninvasive detection of the OSP (Figure 3). The small-diameter, semiround-shaped design concentrates the highest current density at its tip and allows for gentle impression of the electrode into the tissue. This leads to the reduction of the transient resistance between the electrode surface and the targeted nerve, facilitating the delivery of the energy to the target nerve. To increase the penetration of the stimulation impulse through the tissue, a cylindrical magnet was built into the electrodes. The magnetic field creates a tunneling effect, enabling the homogenization and axial direction of the electric field. The synergic combination of the unique shape of the electrode with a built-in magnet allows for nerve excitation using low voltage, thus limiting painful sensations during neuromodulation. The URIS^®^ electrodes are shown in Figure 4.

### 3.3. Biofeedback Foot Sensor (BFS)

The BFS is an accessory of the URIS^®^ device that is attached to the feet of the patient. The BFS contains an analog accelerometer that detects the motor response elicited by every stimulation impulse. The arithmetic mean of the signal amplitude in each of the accelerometer axes is processed by an analog/digital (A/*D*) converter, filtered, and passed to the MCU.

The article "Peroneal Electric Transcutaneous NeuroModulation (eTNM®): A Novel Method for the Treatment of the Overactive Bladder" was published in 2021. Journal: J Healthc Eng.

The localization of the OSP is crucial for achieving the clinical effect of neuromodulation. Based on the information from the BFS confirming the adequate motor response, the MCU determines the precise localization of the OSP at the beginning of each neuromodulation session. Only after the OSP has been confirmed, does the MCU enable initiation of the neuromodulation.

Thanks to the continuous analysis of the data from the BFS, the MCU will adjust the frequency during the neuromodulation session so that the next impulse is enabled only after the motor response to the previous impulse has completely elapsed. This limits muscle fatigue and contributes to the patient's comfort. The intensity of the motor response may vary after a certain period of exposure; therefore, the BFS also allows for continual adjustment of the voltage. This guarantees that the nerve will be permanently exposed to the energy, eliciting the optimal response. Thanks to the closed biofeedback loop, the neuromodulation process is under direct control throughout its duration, as required by the European Union authorities (Medical Devices Regulation 2017/745).

The entire scheme of the URIS^®^ neuromodulation system is shown in Figure 5.

## 4. Materials and Methods

### 4.1. Comparison of the URIS^®^ Electrode versus PTNS Needle and TTNS Self-Adhesive Electrodes

We aimed to compare the URIS^®^ electrode electric output characteristics with those of the electrodes used during PTNS and TTNS in current clinical practice.

We compared the URIS^®^ active electrode to both the L-type needle electrode of diameter 0.23 mm (Seirin, Shizuoka, Japan) and the Stimex^®^ adhesive electrode 50 × 50 mm (Pierenkemper GmbH, Ehringshausen, Germany).

The measurement was performed in a saline-filled vessel in which a neutral electrode of diameter 1 cm was placed 50 mm below the fluid level. Subsequently, all three types of electrodes mentioned above were consecutively inserted into the vessel. The needle electrode was submerged so that its tip was 40 mm below the fluid level. The adhesive electrode floated on the fluid surface, and the hemispherical part of the URIS^®^ electrode was positioned just below the fluid level. All types of active electrodes were consecutively connected to the URIS^®^ device, the output voltage was set to 20 V, the impulse width was 2 ms, and the electric output characteristics were measured.

### 4.2. The Volt-Ampere Characteristics of the Impulses Generated by the URIS^®^ and TTNS Devices

We compared the VA characteristics and other output variables of the URIS^®^ generator with those of the TTNS generator (UROstim2^®^, Schwa-medico GmbH, Ehringshausen, Germany). The measurement was performed as shown in Figure 6. A resistor with a nonload measurement resistance value (100 Ω) was used to measure the current flowing through the circuit. The load was changed for three subsequent measurements: (i) a resistor (*R* = 1 kΩ); (ii) a parallel RC element (*R* = 1000 Ω, *C* = 470 nF) simulating the human body; and (iii) a human volunteer.

The article "Peroneal Electric Transcutaneous NeuroModulation (eTNM®): A Novel Method for the Treatment of the Overactive Bladder" was published in 2021. Journal: J Healthc Eng.

For measurements involving the resistor and RC element, an impulse width of 0.2 ms was used for both generators, representing the standard impulse width for the UROstim2^®^ generator. An output voltage of 15 V was set for the URIS^®^ generator and an output current of 10 mA for the UROstim2^®^ generator.

For measurements involving the human volunteer, the URIS^®^ active electrode and neutral electrode were used. An impulse width of 0.2 ms and the minimal voltage and current values that elicited the motor response of the individual were used (19 V for the URIS^®^ generator and 10 mA for the UROstim2^®^ generator). Subsequently, we performed additional measurement with the URIS^®^ generator set to the standard impulse width of 2 ms and the UROstim2^®^ generator set to the impulse width of 0.4 ms (maximum available impulse width).

### 4.3. Evaluation of Individual Perception of TTNS and Peroneal eTNM^®^

We compared the subjective perception of neuromodulation using several combinations of devices and electrodes using the standard TTNS device UROstim2^®^ and Stimex^®^ electrodes as reference. A total of 14 healthy volunteers (6 males and 8 females) whose average age was 30.9 ± 9.9 years were enrolled. The sequence of stimulations in each individual subject was determined randomly.

For standard Peroneal eTNM^®^ testing, the neutral electrode was placed on the lower abdomen, and the OSP in the popliteal fossa was detected using the URIS^®^ active electrodes. The URIS^®^ device was set at a frequency of 4 Hz and impulse width of 2 ms, and the voltage was then gradually increased until the first motor response was observed. In addition, several measurements were performed as the combination of devices, electrodes, and frequencies was changed.

For the standard TTNS testing, the neutral electrode was placed behind the internal malleolus and the active electrode was placed cranially at approximately 10 cm from the neutral electrode, according to Amarenco [16]. The frequency was set to 10 Hz and the impulse width to 0.2 ms as recommended by the manufacturer. The current intensity was gradually increased until the first motor response was observed.

The article "Peroneal Electric Transcutaneous NeuroModulation (eTNM®): A Novel Method for the Treatment of the Overactive Bladder" was published in 2021. Journal: J Healthc Eng.

After 1 minute of stimulation, the subject was asked to evaluate his/her perception using a visual analog scale (VAS) ranging from 0 (the procedure does not cause me any unpleasant feelings at all) to 100 (the procedure causes me unbearable/unpleasant/painful feelings).

## 5. Results

### 5.1. Comparison of the URIS^®^ Electrode versus PTNS Needle and TTNS Self-Adhesive Electrodes

The measured current intensity was significantly higher than that of the in vivo measurement due to the much lower impedance of saline compared to the human body. At the given output voltage, the measured current and charge values were comparable, while the delivered energy and the current density differed significantly. The needle electrode gave the highest energy and current density. When comparing the noninvasive electrodes, the URIS^®^ electrode delivered 4 times higher energy and 30 times higher current density compared to the Stimex^®^ electrode. These data suggest that the generally recommended standard size self-adhesive surface electrode is not suitable for selective nerve stimulation. Results are summarized in Table 1.

### 5.2. The Volt-Ampere Characteristics of the Impulses Generated by the URIS^®^ and TTNS Devices

When only the resistor was included in the circuit, a rectangular monophasic impulse with a defined width was measured in both generators (Figures 7(a) and 7(b)).

When the RC element was included, there was impulse curve modification due to charging and discharging of the capacitor in both the URIS^®^ and TTNS generators. However, in the TTNS generator, there was a signal overshoot to the opposite polarity caused by connection of the active electrode to the neutral potential of the generator after the impulse had elapsed. This represented the active discharging from the electric RC circuit (Figures 7(c) and 7(d)).

When the human volunteer was included in the circuit as a load, an approximately constant voltage was measured over the duration of the impulse with the URIS^®^ generator and a constant current over the duration of the impulse with the TTNS generator.

In case of URIS^®^, there was a change in current flowing through the patient during the impulse duration. In the first few microseconds of the impulse, a peak current corresponding to the charge required for stimulation was delivered into the patient's body. This current value decreased during the impulse duration, due to the required charge, which was determined as

(1) $$\begin{array}{c} Q=I\cdot t, \end{array}$$

where *I* represents the current intensity and *t* represents the impulse width.

Based on the impulse character, the charge was determined as

(2) $$\begin{array}{c} Q=\int_{0}^{t}I\text{d}t\\ =\int_{0}^{t}U\cdot R\text{d}t, \end{array}$$

where *I* represents the current intensity, *U* represents the voltage, *R* represents the resistance, and *t* represents the impulse width.

The article "Peroneal Electric Transcutaneous NeuroModulation (eTNM®): A Novel Method for the Treatment of the Overactive Bladder" was published in 2021. Journal: J Healthc Eng.

Due to the short peak of the current pulse, a substantial proportion of the required charge was supplied during the initial part of the impulse, and subsequently, this charge was kept almost constant. This approach prevented long exposure of the patient to the large charge. As soon as the impulse elapses, the URIS^®^ generator immediately disconnects the patient electronically from the circuit, allowing for the remaining voltage to naturally discharge from the body (Figure 8(a)).

When the TTNS generator was used, an electric charge was supplied to the patient throughout the impulse duration, which constantly increased over the impulse duration. Once the impulse elapses, the output of the TTNS generator is automatically switched to the neutral potential of the generator, which causes active discharge of the current accumulated in the body. This is reflected in the biphasic current curve, where the peak current intensity flowing through the patient's body during discharging is several times higher than that originally generated, which could be painful to the patient and may attenuate the clinical efficacy (Figure 8(b)). The monophasic VA curve demonstrates the absence of active discharging of the patient's body when using the URIS^®^ generator at an impulse width of 0.2 ms (Figure 8(c)).

When evaluating the amount of energy and charge delivered to the body during stimulation with an impulse of width 0.2 ms by the URIS^®^ and UROstim2^®^ generators, we did not observe any significant difference. The energy supplied to the human body when a 2 ms impulse was generated by URIS^®^ was significantly higher but still reduced the patient's exposure, that is, the current and voltage passing through the body. The impulse width extension using the UROstim2^®^ device resulted in a significant increase in the voltage, while the extension of the impulse width using the URIS^®^ device led to a reduction of the voltage and current required for effective nerve stimulation. This results in a significant reduction in exposure to the patient and limits potential risk (Table 2).

### 5.3. Evaluation of Individual Perception of TTNS and Peroneal eTNM^®^

The average VAS score was 34.8 ± 17.4 for standard TTNS, 66.3 ± 12.5 for peroneal stimulation using the combination of Stimex^®^ electrodes and UROstim2^®^ device, and 13.8 ± 16.5 for standard Peroneal eTNM^®^. When stimulating the peroneal nerve using Stimex^®^ electrodes, the VAS score was significantly higher than that for the standard Peroneal eTNM^®^, regardless of the device and frequency combination used. The results of all measured variables are summarized in Table 3.

The article "Peroneal Electric Transcutaneous NeuroModulation (eTNM®): A Novel Method for the Treatment of the Overactive Bladder" was published in 2021. Journal: J Healthc Eng.

### 5.4. Early Clinical Experience

The following case reports refer to the first consecutive patients treated using Peroneal eTNM^®^ rather than preselected successfully treated responders. These reports demonstrate the impact of OAB on patient-reported quality of life. It is obvious that an evaluation of the efficacy and safety of the Peroneal eTNM^®^ awaits the results of standard clinical studies.

All presented patients were considered nonresponders to the previous behavioral and pharmacological OAB therapies. All patients were significantly bothered by persistent OAB symptoms and sought further treatment. All patients provided informed consent. Treatment using Peroneal eTNM^®^ was approved by both the Institutional Ethics Committee and Scientific Board of the University Hospital, Motol, Prague.

All patients were treated in outpatient settings in 30-minute sessions, once a week for 12 weeks. The frequency was 4 Hz, impulse width was 2 ms, and the voltage was set individually to the lowest value that elicited a motor response.

#### 5.4.1. Case 1: M. K. (a 72-Year-Old Female)

This patient, with a history of hypertension, metabolic syndrome (BMI 43), and abdominal hysterectomy due to benign condition, had been suffering from OAB symptoms for 2 years. Previous treatment using several anticholinergics and betamimetics failed due to adverse events. According to the 3-day bladder diary, the patient reported 7 episodes of micturition per day before Peroneal eTNM^®^ treatment. The most bothersome issues for her were 2 episodes of severe urgency per day when she had to rush to the toilet, and additional 1-2 episodes of urgency incontinence per day, when she suffered urine leak before reaching the toilet. These symptoms significantly limited her social activities, and she left home only on rare occasions. After Peroneal eTNM^®^ treatment, the micturition frequency remained unchanged, but episodes of severe urgency and urgency incontinence completely disappeared. The warning time from the first sensation of urgency to voluntary micturition increased significantly. She did not notice any side effects during the treatment and marked her health condition as very much improved on the Likert scale.

#### 5.4.2. Case 2: T. Z. (a 30-Year-Old Female)

This patient, an otherwise healthy woman with a history of OAB since childhood (over 20 years), had been previously treated with several anticholinergics without any notable effect. After the treatment trial with betamimetics, the patient observed a partial reduction in symptoms but did not consider this sufficient. Therefore, she was referred for treatment with Peroneal eTNM^®^. According to the 3-day bladder diary, the patient had an average of 17 episodes of micturition per day at baseline. Ten of those were preceded by severe urgency. The urodynamic assessment revealed the bladder oversensitivity during filling cystometry. After Peroneal eTNM^®^ treatment, the micturition frequency was reduced to 11 per day (−67% considering the frequency of 8 episodes of micturition per day to be normal) and the number of severe urgency episodes was reduced to 3 per day (−70%). The patient reported significant improvement in her bladder condition by 2 points, as documented by the 6-point Patient Perception of the Bladder Condition (PPBC) scale.

The article "Peroneal Electric Transcutaneous NeuroModulation (eTNM®): A Novel Method for the Treatment of the Overactive Bladder" was published in 2021. Journal: J Healthc Eng.

#### 5.4.3. Case 3: K. L. (a 54-Year-Old Female)

This patient had a history of multiple sclerosis diagnosed in 2012, which was later classified as a relapsing-remitting course; she had been treated with interferon and subsequently with fingolimod. The expanded disability status scale (EDSS) score was 5.0/10.0.

The patient was referred to a urologist due to OAB symptoms she had suffered for 4 years. Initial treatment attempt with betamimetics was not effective and the patient was subsequently suggested for Peroneal eTNM^®^. At the baseline, the patient was bothered by an average of 16.3 episodes of micturition, 2.7 episodes of severe urgency, and 0.7 episodes of urgency incontinence per day, as reported in her 3-day bladder diary. A reduced cystometric capacity (230 mL), normal compliance, and terminal detrusor overactivity (maximum detrusor pressure of 37 cm H_2_O) were documented during filling cystometry, while the voiding phase was not impaired with complete emptying. After Peroneal eTNM^®^ treatment, the micturition frequency decreased to an average of 10 episodes per day (−76% considering the frequency of 8 episodes of micturition per day to be normal) and the number of severe urgency episodes reduced to 1.0 per day (−71%). The patient reported complete disappearance of urgency incontinence and a significant reduction in nocturia episodes from 2.7 to 0.7 (−74%). This contributed to the reduction of her chronic fatigue and allowed for an increase in her daily activity. The patient reported significant improvement in her bladder condition by 2 points as documented by the PPBC scale.

## 6. Discussion

OAB syndrome is a chronic medical condition with a proven detrimental impact on QoL and well-documented health consequences for affected individuals [17]. Its treatment goals include maximizing symptom control and QoL while minimizing adverse events [18]. There is a wide range of OAB treatment methods available, but neither of these represents an ideal therapeutic tool. All currently existing methods are associated with certain drawbacks, which limit their wide use in clinical practice. Given the high prevalence of OAB and its burden on both individuals and societies, the development of a long-term effective, safe, and easy-to-use treatment method is highly desirable.

The article "Peroneal Electric Transcutaneous NeuroModulation (eTNM®): A Novel Method for the Treatment of the Overactive Bladder" was published in 2021. Journal: J Healthc Eng.

The selective stimulation of the peroneal nerve using the URIS^®^ device has a number of advantages. The course of the peroneal nerve makes it possible to precisely define the OSP. Exact localization of this small area in the popliteal fossa is a prerequisite for eliciting an adequate motor response. Determination of the OSP based on both the sensation and visible motor response (mediolateral feet movement) represents a fundamental difference compared to the TTNS method, in which the OSP is not clearly defined. Some authors recommend placing the active electrode approximately 5–10 cm above the inner ankle, while others recommend placing it just posterior to the inner ankle [19, 20]. In some TTNS devices, the differentiation between the active and neutral electrodes is missing, which can be confusing while placing the electrodes. Due to a lack of standardization of electrode positions, the response to TTNS may vary widely, from a slight tingling sensation felt on the sole of the foot through the flexion of the thumb to the flexion of all toes. Sometimes patients wrongly consider a throbbing or burning sensation under the electrode or a stinging sensation in the calf, arising from the conduction of current in the superficial veins, to be an adequate response to the TTNS stimulation.

There are several technical features of the URIS^®^ device to be pointed out. The URIS^®^ device represents a constant voltage source with current intensity decreasing over the impulse duration. The electrical disconnection of the patient from the URIS^®^ generator after the impulse has subsided warrants that the patient is not exposed to any additional current flow. Other features that contribute to patient safety are galvanic separation of the patient and the presence of a voltage boost converter that cuts off the patient's exposure to the voltage in the event of a hardware or firmware failure. The entire design of the URIS^®^ device makes it possible to achieve a clinical effect at a significantly lower voltage and current compared to the currently used TTNS devices which are designed as current generators.

One of the major advantages of the URIS® system has to do with the URIS® active electrodes. The human body is considered a conductor of the II type because the electric current is conducted in the body by ions. The most significant change in the electric field compared to a homogeneous medium occurs in the skin, which is responsible for more than 99% of the body's resistance to the electric current flow [21]. The vast majority of the electric current passes through the skin barrier by means of the sweat glands. Ohmic and capacitive impedance of the skin limits the depth of penetration of the electric impulse. The hemispherical shape of the URIS^®^ electrodes allows for high current density at the tip of the electrode and for its gentle impression into the tissue, reducing the resistance. These facts, along with impulse modulation by the magnetic field, enable selective nerve stimulation without simultaneous excitation or irritation of the surrounding structures, including the nociceptive receptors in the skin and subcutaneous tissue, thus reducing the unpleasant and painful sensations during the neuromodulation. Compared to the standard self-adhesive electrodes routinely used in TTNS, a much lower impulse intensity is required to deliver the same energy to the target nerve even in obese patients, where the distance between the electrode and the peroneal nerve is longer due to fat tissue deposits. Based on the laboratory testing, the effect of the URIS^®^ electrode is close to that of the needle electrode, without the need to compromise the skin integrity. In addition, presented data on treatment perception show that the URIS^®^ electrodes, which are an integral part of the URIS^®^ neuromodulation system, cannot be replaced by any type of self-adhesive surface electrodes used in TTNS.

The article "Peroneal Electric Transcutaneous NeuroModulation (eTNM®): A Novel Method for the Treatment of the Overactive Bladder" was published in 2021. Journal: J Healthc Eng.

The incorporation of the biofeedback loop into the URIS^®^ system represents another significant advantage. The BFS allows for precise localization of the OSP and ensures that the treatment session does not start until the optimal position of the active electrode has been achieved. After the neuromodulation has been initiated, based on the feedback data, the MCU will continuously adjust the voltage and frequency in order to keep the output energy as high as necessary for effective neuromodulation and as low as possible to prevent side effects. The URIS^®^ system software records and stores the retrospective data on impulse voltage, impulse frequency, and number and length of individual neuromodulation sessions that the patient has completed. With its noninvasiveness and biofeedback features, the URIS^®^ system is compatible with the FDA and EU regulations for home-based use. The device is able to check the patient's adherence and, if necessary, reminds the patient of the correct treatment schedule. The URIS^®^ system allows the physician to share the patients' data on treatment progress and change the stimulation parameters or treatment schedule as needed using remote access. This technology ensures that, even in home-based use, the treatment can be fully under professional control and continuously modified in order to achieve the optimal therapeutic effect.

The article "Peroneal Electric Transcutaneous NeuroModulation (eTNM®): A Novel Method for the Treatment of the Overactive Bladder" was published in 2021. Journal: J Healthc Eng.

PTNS is considered the standard peripheral neuromodulation method currently used in OAB treatment. The use of the needle electrode represents its most significant limitation. The placement of the electrode tip in the proximity of the tibial nerve can be challenging and may be associated with uncomfortable sensations or pain. Transcutaneous electrical nerve stimulation (TENS) has been used in pain treatment since the end of the 1960s [22]. The mechanism of action of TENS is not fully elucidated, but it is thought to include the release of endogenous opioids and blocking of the nociceptive stimuli by activation of nonpainful sensations, according to the gate control theory by Melzack [23]. The TENS technique with surface electrodes located over the tibial nerve course, referred to as TTNS, was first used for OAB treatment in the 1990s [24]. Although TTNS and Peroneal eTNM^®^ may seem to be similar, these two methods differ in principle. While Peroneal eTNM^®^ is based on selective stimulation of the nerve with minimal excitation of other sensory receptors, TTNS produces stimulation over a large area of the skin surface, which, according to the gate control theory, can cause blocking of a certain proportion of the afferent stimuli at the level of the synapsis between the primary and secondary neurons. This may attenuate its clinical efficacy. In addition, there are a number of other factors that distinguish Peroneal eTNM^®^ from TTNS. Our data show that, due to the combination of several original technical innovations, including different generator constructions with unique impulse patterns and effective URIS^®^ electrodes, Peroneal eTNM^®^ is much better perceived than TTNS. Its noninvasiveness and use of the biofeedback control make Peroneal eTNM^®^ easy to use by patients themselves in their home environment without any assistance.

During the clinical testing, we were able to demonstrate that Peroneal eTNM^®^ may represent a feasible method for OAB treatment. In a small cohort of patients with OAB, we observed a significant reduction in OAB symptoms, as demonstrated using standardized tools in response to Peroneal eTNM^®^. At the same time, we did not observe any adverse event during the treatment. Although these preliminary results are encouraging, they need to be confirmed by large well-designed prospective clinical trials.

The article "Peroneal Electric Transcutaneous NeuroModulation (eTNM®): A Novel Method for the Treatment of the Overactive Bladder" was published in 2021. Journal: J Healthc Eng.

## 7. Conclusion

Peroneal eTNM^®^ using the URIS^®^ neuromodulation system represents a new method for the treatment of OAB symptoms. It boasts unique features that differentiate it significantly from other currently available neuromodulation techniques. Further well-designed prospective clinical trials are required to assess its efficacy and safety.

## Figures and Tables

**Figure 1:** URIS^®^ active electrode position on the skin in the popliteal fossa and the peroneal nerve course. The magnetic resonance (MR) scan demonstrating the URIS^®^ active electrode (for the MR imaging purposes, the electrode was replaced by a wet cotton swab) marked with a white arrow located in the immediate vicinity of the peroneal nerve (marked with the black arrow).

**Figure 2:** The optimal stimulation point (OSP) used for Peroneal eTNM^®^ in the popliteal fossa. The OSP (marked in black) is determined by eliciting a typical sensation and visible motor response in terms of rhythmic movement of the foot using the output voltage of 20 V. The dotted line represents an area where the sensitive response, but not motor response, can be elicited. The precise location of the OSP may vary and needs to be determined individually in every patient before the neuromodulation is initiated.

**Figure 3:** The scheme of the URIS^®^ active electrode (1: silver-plated electrode surface; 2: permanent magnet; 3: diamagnetic part; 4: conductive part of the electrode; 5: electrode top cover).

**Figure 4:** The URIS^®^ active and neutral electrodes. The URIS^®^ active electrode searching for the optimal stimulation point at the popliteal fossa (a). Self-adhesive neutral electrode attached to the lower abdomen (b).

**Figure 5:** Block wiring diagram of the URIS^®^ neuromodulation system (BFS: biofeedback foot sensor; MCU: microcontroller unit; A/D converter: analog/digital converter).

**Figure 6:** Wiring diagram of the circuit used to compare volt-ampere (VA) characteristics of stimulation impulses generated by URIS^®^ and TTNS devices. The resistor with a nonload measurement resistance value (100 Ω) was used to measure the current flowing through the circuit (VB). The total output signal from the generators is measured between the output terminals (VA). The load was changed for three subsequent measurements: (i) resistor (*R* = 1kΩ), (ii) parallel RC element simulating the human body (*R* = 1000 Ω and *C* = 470 nF), and (iii) a human volunteer.

**Figure 7:** The volt-ampere characteristics of the impulses generated by the URIS^®^ and TTNS generators using a resistor and parallel RC element as a load. Impulse shape with a resistor (*R* = 1 kΩ) as measured using the URIS^®^ (a) and TTNS (b) generators. Impulse shape with a parallel RC element simulating the human body (*R* = 1000 Ω and *C* = 470 nF) as measured using URIS^®^ (c) and TTNS (d) generators. The URIS^®^ active electrode was used for all measurements. Setting parameters: impulse width of 0.2 ms, output voltage of 15V  for the URIS^®^ generator, and output current of 10 mA for the TTNS generator.

The article "Peroneal Electric Transcutaneous NeuroModulation (eTNM®): A Novel Method for the Treatment of the Overactive Bladder" was published in 2021. Journal: J Healthc Eng.

**Figure 8:** The volt-ampere characteristics of the pulses generated by the URIS^®^ and TTNS generators using a human body as a load. Impulse shape with the human body as a load as measured using the URIS^®^ (a) and TTNS (b) generators. The URIS^®^ active electrode was used for all measurements. Setting parameters: impulse width of 0.2 ms, output voltage of 19 V for the URIS^®^ generator, and output current of 10 mA for the TTNS generator. Impulse shape with the human body as a load as measured using the URIS^®^ generator (c). The URIS^®^ active electrode was used. Setting parameters: impulse width of 2 ms and output voltage of 15 V.

**Table 1:** The electric output characteristics of various electrodes used for peripheral neuromodulation.

	Current (mA)	Charge (*µ*C)	Energy (mJ)	Square (mm^2^)	Current density (mA/mm^2^)
L-type needle electrode	43.4	72.0	0.6	28.9	1.503
URIS^®^ active electrode	45.8	68.0	0.4	94.5	0.484
Stimex^®^ self-adhesive electrode	38.4	74.0	0.1	2500.0	0.015

All types of active electrodes were consecutively connected to the URIS^®^ device, the output voltage was set to 20 V, and the impulse width was 2 ms. The data show that the needle electrode provided the highest energy and current density. Comparing the noninvasive electrodes, the URIS^®^ electrode provided 4 times higher energy and 30 times higher current density compared to the Stimex^®^ adhesive electrode.

**Table 2:** The volt-ampere characteristics of the impulses generated by the URIS^®^ and UROstim2^®^ generators when the human volunteer was included in the circuit as a load.

Device	UROstim2^®^	UROstim2^®^	URIS^®^	URIS^®^
Electrodes	URIS^®^	URIS^®^	URIS^®^	URIS^®^
Impulse width (ms)	0.2	0.4	0.2	2.0
Voltage (V)	30.3	42.0	18.9	15.0
Current (mA)	10.0	9.6	11.9	4.3
Energy (mJ)	0.066	0.161	0.044	0.130
Charge (*µ*C)	2.0	3.8	2.4	8.6

The voltage and current are presented as RMS values. The data demonstrate that extending the impulse width using the UROstim2^®^ device led to a significant increase in voltage, while extending the impulse width using the URIS^®^ device led to a reduction of the voltage and current required for effective nerve stimulation. This results in a significant reduction in exposure to the patient.

**Table 3:** Individual perception of neuromodulation using different combinations of the URIS^®^ and UROstim2^®^ generators and electrodes.

	Peroneal nerve				Tibial nerve
Device	URIS^®^	URIS^®^	UROstim2^®^	UROstim2^®^	UROstim2^®^
Electrodes	URIS^®^	Stimex^®^	Stimex^®^	Stimex^®^	Stimex^®^
Impulse width (ms)	2.0	2.0	0.2	0.2	0.2
Frequency (Hz)	4.0	4.0	4.0	10.0	10.0
Voltage (V)	22.2 ± 6.2	59.3 ± 17.0	52.2 ± 13.7	49.2 ± 14.1	62.5 ± 23.7
Current (mA)	6.8 ± 1.4	34.9 ± 10.0	43.5 ± 11.4	41.0 ± 11.8	27.8 ± 7.1
Energy (mJ)	0.2 ± 0.1	0.4 ± 0.3	0.5 ± 0.2	0.4 ± 0.2	0.3 ± 0.2
VAS	13.8 ± 16.5	83.8 ± 11.1	56.3 ± 7.5	66.3 ± 12.5	34.8 ± 17.4

The data demonstrate that the standard Peroneal eTNM^®^ uses a significantly lower impulse intensity and is associated with significantly less discomfort compared to the standard TTNS. VAS: visual analog scale.

The article "Peroneal Electric Transcutaneous NeuroModulation (eTNM®): A Novel Method for the Treatment of the Overactive Bladder" was published in 2021. Journal: J Healthc Eng.

## Data Availability

The datasets used and analysed during the current study are available from the corresponding author upon reasonable request.
